# SBP-0636457, a Novel Smac Mimetic, Cooperates with Doxorubicin to Induce Necroptosis in Breast Cancer Cells during Apoptosis Blockage

**DOI:** 10.1155/2022/2390078

**Published:** 2022-07-11

**Authors:** Rui Yu, Lei Wang, Xiaochun Ji, Chenxiao Mao

**Affiliations:** ^1^Department of Biochemistry, School of Medicine, Ningbo University, Ningbo, Zhejiang, China; ^2^Department of Electronic Commerce, Zhejiang Fashion Institute of Technology, Ningbo, Zhejiang, China

## Abstract

Breast cancer (BC) is a common health concern worldwide. Doxorubicin (Dox) is a widely used chemotherapeutic agent to treat various cancers, including BC. However, drug resistance and severe side effects often hinder the clinical application of Dox. Combination therapy is an effective potent strategy to increase chemosensitivity and reduce the adverse effects. Smac is a proapoptotic protein that interacts with inhibitors of apoptosis proteins (IAPs) and thereby promotes cell death. Smac mimetic compounds can mimic its function and can be used to kill cancer cells. In this study, Dox and SBP-0636457, a novel Smac mimetic, were found to have cooperative effects in inducing BC cell death. Dox and SBP-0636457 cotreatment induced necroptosis instead of apoptosis in BC cells. Receptor-interacting serine/threonine-protein kinase 1 or mixed-lineage kinase domain-like silencing could attenuate cell death caused by Dox/SBP-0636457 in BC cells. In addition, this combined treatment caused synergistic induction of TNF*α*, and TNF*α*/TNFR signalling is essential for cell death induced by Dox/SBP-0636457 in BC cells. Moreover, both canonical and noncanonical nuclear factor kappa B pathways were found to contribute to TNF*α* upregulation induced by Dox/SBP-0636457. Therefore, the findings suggest that SBP-0636457 combined with Dox is an alternative strategy for treating BC.

## 1. Introduction

Breast cancer (BC) is a common type of cancer and a leading cause of cancer-related deaths among women worldwide [1]. Although its treatment greatly advanced in the past decades, the overall survival of patients with BC remains unsatisfactory [2]. Currently, chemotherapy remains a backbone treatment for BC, especially in patients at an advanced stage. Doxorubicin (Dox), also known as Adriamycin, is the most effective anticancer and chemotherapeutic agent for the treatment of BC [3]. However, resistance to Dox remains a major clinical barrier and prevents its clinical application. Increasing evidence suggests that Dox resistance is mainly caused by apoptotic evasion, a well-investigated form of programmed cell death (PCD). Therefore, effective combination treatment of Dox with other agents should be identified to overcome drug resistance.

Necroptosis, another form of PCD, is morphologically and mechanistically different from apoptosis [4] because it is activated by a unique caspase-independent signalling pathway and promotes the formation of the RIPK1/RIPK3/mixed-lineage kinase domain-like (MLKL) complex [5]. Recent studies have reported that triggering necroptosis may be a potent treatment strategy to kill cancer cells, especially those resistant to apoptosis [6].

Smac is a proapoptotic protein that is released from the mitochondria by activating the intrinsic apoptotic pathway [7]. It can antagonise the cellular inhibitor of the apoptosis protein (IAP) family that negatively regulates the cell death process [8]. IAP proteins inhibit cell death by modulating the nuclear factor kappa B (NF-*κ*B) signalling pathway [8]. IAP upregulation has been found in various cancers and is correlated with the poor prognosis of BC. Therefore, synthetic Smac mimetics can induce IAP ubiquitination and degradation and evaluate various cancers [9]. For instance, a designed Smac mimetic (SM-131,2) can effectively antagonise XIAP, a member of IAPs, and induce apoptosis in BC cells [10]. Another Smac mimetic ARTS promoted BC cell death by inducing XIAP degradation [11].

SBP-0636457 is a novel Smac mimetic. To date, knowledge regarding the effects of SBP-0636457 on cancer cells has been limited. The present study demonstrated that SBP-0636457 and Dox cotreatment can induce BC cell death. Investigation of the underlying mechanisms indicated that SBP-0636457 and Dox trigger necroptosis instead of apoptosis in BC cells. The findings suggest that SBP-0636457 combined with Dox is an effective treatment for BC, especially in the case of insensitivity to apoptosis.

## 2. Materials and Methods

### 2.1. Reagents and Antibodies

SBP-0636457 was obtained from MedChemExpress (USA). SBP-0636457 was dissolved in sterile DMSO at the concentration of 5 mM and kept at −80°C. Dox, Nec-1, RIP-56, GSK481, MLKL-IN-1, and GW806742X were purchased from Selleck Chemicals (USA). z.VAD, PS-341, QNZ, and Enbrel were purchased from Sigma-Aldrich (USA). The following antibodies obtained from CST antibodies (USA) were used: anti-caspase-8 (cat: 9746; dilution: 1:1000), anti-Fas-associated death domain (FADD) (cat: 9746; dilution: 1:1000), anti-receptor-interacting serine/threonine-protein kinase 1 (RIP1) (cat: 98110; dilution: 1:1000), MLKL (cat: 37705; dilution: 1:1000), TNFR1 (cat: 3736; dilution: 1:1000), p65 (cat: 3033; dilution: 1:1000), and NIK (cat: 4994; dilution: 1:1000). The GAPDH (cat: 9001-50-7; dilution: 1:5000) and HRP conjugate secondary antibodies (cat:12-348; dilution: 1:4000) were purchased from Sigma-Aldrich.

### 2.2. Cell Culture

Human BC cells (MDA-MB-231, MCF-7, MDA-MB-453, and Hs578T) were purchased from ATCC (USA) and were cultured in the RPMI1640 medium (Gibco, USA) supplemented with 10% foetal bovine serum (FBS, Life Technologies) and 100 units/ml penicillin/streptomycin (Sigma) in a cell culture incubator at 37°C and 5% CO_2_.

### 2.3. Cell Death Measurement

Cell death was measured using the Annexin V-FITC/PI detection kit (BD Biosciences, USA) following the manufacturer's guide. To measure the cell death induced by SBP-0636457, BC cells were treated with various doses of SBP-0636457 (0.5 *μ*M, 1 *μ*M, 1.5 *μ*M, 2, 5 *μ*M) for 24 h. To assess the effects of various cell death inhibitors, cells were cotreated with SBP-0636457 and different cell death inhibitors for 24 h. Then, cells were harvested and washed with an ice-cold paraffin-based solution. Thereafter, the cells were incubated with staining buffer containing annexin V-FITC/PI for 20 min in the darkroom at room temperature. Flow cytometry was performed (BD Bioscience, USA), and data were analysed using FlowJo software.

### 2.4. RNA Interference

Cells were transfected with siRNA oligos using Lipofectamine 2000 (Life Technologies, USA) according to the manufacturer's guide. The siRNA oligos were synthesised by GenePharma Ltd (China). The siRNA oligo sequences are listed in Table 1.

### 2.5. RNA Isolation and Quantitative Polymerase Chain Reaction (qPCR)

After different treatments, cells were collected, and the total RNA was extracted using Trizol Reagent (Life Technologies) following the manufacturer's instructions. Thereafter, the total RNA was reverse transcribed to cDNA using the RevertAid First Strand cDNA synthesis kit (Thermofisher, USA). For the quantification of gene expression, SYBR green-based quantitative real-time PCR (Applied Biosystems, USA) was performed using the QuantStudio Real-Time PCR system (Applied Biosystems). The primers used are listed in Table 2.

### 2.6. Western Blotting

After treatment, cells were collected and lysed using the RIPA lysis buffer (Beyotime, China). Thereafter, equal amounts of proteins were loaded onto 12% SDS-PAGE and subjected to electrophoresis. Subsequently, the proteins were transferred onto a PVDF membrane and incubated with primary antibodies overnight at 4°C, followed by incubation with the corresponding secondary antibodies for 1 h at room temperature. Most western blotting was conducted by an experimenter who was blinded to the samples.

### 2.7. Statistical Analysis

Statistical analyses were performed using SPSS 12.0 (IBM, Chicago, IL, USA). Data were expressed as the mean ± standard deviation. Student's *t*-test (two-tailed distribution, two-sample, and unequal variance) was used for between-group comparisons, and a one-way analysis of variance, followed by Tukey's post hoc test, was used for comparing multiple groups. A *P* value of <0.05 (two-tailed) was considered statistically significant.

## 3. Results

### 3.1. Combined Treatment with SBP-0636457 and Dox Can Induce BC Cell Death

Four different BC cells (MDA-MB-231, MCF7, MDA-MB-453, and Hs578T) were treated with various doses of SBP-0636457 for 24 h, and cell death was measured. SBP-0636457 was found to induce cell death in a dose-dependent manner (Figure 1(a)). Therefore, to identify the form of cell death induced by SBP-0636457, a specific apoptosis inhibitor (z.VAD) was used. Interestingly, z.VAD was found to promote cell death induced by SBP-0636457 (Figure 1(b)). The combined effect was also observed, and only a slight difference was observed between the combined treatment of SBP-0636457 and Dox and of SBP-0636457 alone (Figure 1(b)). However, SBP-0636457/Dox/z.VAD induced more cell death than SBP-0636457/Dox in BC cells (Figure 1(b)). Interestingly, Nec-1, a specific RIPK1 inhibitor, was found to significantly reduce cell death induced by SBP-0636457/Dox/z.VAD in BC cells (Figure 1(b)). This finding points towards the RIPK1-dependent necroptotic cell death. Thereafter, we measured the levels of some essential proteins involved in cell death (Figure 1(c)). Because z.VAD-mediated apoptotic inhibition only mimics apoptotic resistance partially and in a relatively artificial manner, siRNAs were used to knock down caspase-8 or FADD in BC cells to mimic apoptotic resistance (Figure 1(d)). In addition, silencing of either caspase-8 or FADD could markedly increase cell death induced by SBP-0636457/Dox (Figures 1(e), 1(f)). These findings confirmed the effects observed in SBP-0636457/Dox/z.VAD-treated cells and excluded the potential side effects of z.VAD. Therefore, the results suggest that SBP-0636457 combined with Dox induces necroptosis in BC cells but inhibits apoptosis.

### 3.2. SBP-0636457/Dox Induces Cell Death in a RIPK1- and MLKL-dependent Manner in BC Cells

The kinase RIPK1 is an important regulator of necroptosis [12]. Therefore, we evaluated its role in the cell death caused by SBP-0636457/Dox/z.VAD in BC cells. Two siRNAs were used to successfully knock down RIPK1 in BC cells (Figure 2(a), left), which found that silencing of RIPK1 markedly reduced cell death caused by SBP-0636457/Dox/z.VAD in BC cells (Figure 2(b)). To further assess whether RIPK1 is required for cell death induced by SBP-0636457/Dox/z.VAD, two RIPK1 inhibitors (RIPA-56 and GSK481) were used. Both RIPA-56 and GSK481 were found to significantly reduce the cell death induced by SBP-0636457/Dox/z.VAD (Figure 2(c)). Because MLKL is another necroptosis regulator and has been found to interact with RIPK1 [12], its role in cell death induced by SBP-0636457/Dox/z.VAD was also examined. Two siRNAs were used to inhibit MLKL expression in BC cells (Figure 2(a), right), and the results revealed that cell death induced by SBP-0636457/Dox/z.VAD markedly reduced after MLKL knockdown in BC cells (Figure 2(d)). Subsequently, two MLKL inhibitors (MLKL-IN-1 and GW806742X) were used, which significantly decreased cell death induced by SBP-0636457/Dox/z.VAD in BC cells (Figures 2(e), 2(f)). Therefore, these results suggest that RIPK1 and MLKL are required for cell death induced by SBP-0636457/Dox/z.VAD in BC cells.

### 3.3. TNF*α*/TNFR/IRF1 Signalling Is Required for Cell Death Induced by SBP-0636457/Dox

Previous studies have suggested that TNF*α* plays an essential role in necroptosis [13]. Therefore, the effects of SBP-0636457/Dox on TNF*α*/TNFR signalling were examined in this study. TNF*α* secretion in the supernatant was measured using the enzyme-linked immunosorbent assay (ELISA). Dox or SBP-0636457 treatment alone was found to slightly induce TNF*α* upregulation (Figure 3(a)). In addition, TNF*α* upregulation was higher after combined treatment with Dox/SBP-0636457 than after treatment with either of these agents alone (Figure 3(a)). RT-PCR results also showed that upregulation of TNF*α* mRNA was higher after Dox and SBP-0636457 cotreatment than after treatment with either of these agents alone (Figure 3(b)). To examine the role of TNF*α* in necroptosis induced by SBP-0636457/Dox, the TNF*α*-blocking antibody Enbrel was used, which significantly reduced cell death induced by SBP-0636457/Dox (Figure 3(c)). Furthermore, siRNAs were used to knock down TNFR in BC cells (Figure 3(d), left), and the results revealed that TNFR silencing markedly reduced cell death induced by SBP-0636457/Dox/z.VAD in BC cells (Figure 3(e)). Moreover, IRF1 is a transcription factor that can be induced by TNF*α* and plays an essential role in necroptosis induced by Smac mimetics. Therefore, IRF1 expression after SBP-0636457/Dox treatment was also examined. RT-PCR showed that combined treatment with SBP-0636457 and Dox markedly upregulated IRF1 mRNA in BC cells (Figure 3(f)). To investigate the role of IRF1 in cell death induced by SBP-0636457/Dox, siRNAs against IRF1 were used in BC cells (Figure 3(g)), and it was found that IRF1 silencing markedly reduced cell death induced by SBP-0636457/Dox/z.VAD in BC cells (Figure 3(h)). Altogether, these results suggest that TNF*α*/TNFR/IRF1 signalling is required for necroptosis induced by SBP-0636457/Dox/z.VAD in BC cells.

### 3.4. Both Canonical and Noncanonical NF-ΚB Pathways Contribute to TNF*α* Upregulation after SBP-0636457/Dox Treatment

The mechanisms underlying TNF*α* upregulation after SBP-0636457/Dox treatment were investigated because the NF-*κ*B pathway is reported to be involved in TNF*α* upregulation [14]. However, whether the NF-*κ*B pathway is responsible for the cell death induced by SBP-0636457/Dox/z.VAD remains to be elucidated. Two siRNAs were used to knock down the NF-*κ*B subunit p65, a key component of the canonical NF-*κ*B pathway (Figure 4(a)). p65 silencing only partially reduced cell death induced by SBP-0636457/Dox/z.VAD (Figure 4(b)). Therefore, the involvement of the noncanonical NF-*κ*B pathway was further investigated by analysing the stabilisation of NIK protein, a key upstream kinase involved in the noncanonical NF-*κ*B pathway. NIK accumulation was observed within 2 h of SBP-0636457/Dox treatment in BC cells (Figure 4(c)). Thereafter, siRNAs were used to knock down NIK in BC cells (Figure 4(d)). NIK inhibition only partially reduced cell death induced by SBP-0636457/Dox/z.VAD in BC cells (Figure 4(b)). Based on these findings, siRNAs were used to inhibit both p65 and NIK, which reduced cell death caused by SBP-0636457/Dox/z.VAD more effectively than that caused by inhibition of either p65 or NIK (Figure 4(b)). In addition, upregulation of TNF*α* mRNA induced by SBP-0636457/Dox/z.VAD was reduced after p65 and NIK inhibition compared with silencing of p65 or NIK alone in BC cells (Figure 4(e)). Furthermore, the canonical NF-*κ*B inhibitor NG25 and noncanonical NF-*κ*B inhibitor NIK SMI1 reduced cell death to a lesser extent than the dual NF-*κ*B inhibitor DHMEQ (Figure 4(f)). Compared with the dual NF-*κ*B inhibitor NG25 or NIK SMI1, DHMEQ reduced TNF*α* mRNA upregulation (Figure 4(g)). Therefore, these findings suggest that both canonical and noncanonical NF-*κ*B promote necroptosis and TNF*α* upregulation induced by SBP-0636457/Dox in BC cells.

## 4. Discussion

BC is one of the primary public health issues worldwide and is commonly treated with chemotherapy, surgery, and radiotherapy. However, dysregulation of apoptosis-related proteins frequently causes drug resistance and decreases the therapeutic efficacy [15]. Therefore, targeting necroptosis, another form of PCD, represents an alternative strategy to kill cancer cells. In recent years, several studies have suggested that Smac mimetics can induce necroptosis in various cancer cells alone or combined with other agents. In the present study, SBP-0636457, a novel Smac mimetic, was found to cooperate with Dox to induce necroptosis in BC cells. Mechanically, RIPK1 and MLKL are essential for necroptosis induced by SBP-0636457/Dox in BC cells. Furthermore, SBP-0636457/Dox activates the NF-*κ*B/TNF*α*/TNFR/IRF axis and is also required to induce necroptosis.

Several studies have shown that Dox and Smac mimetics showed synergistic antitumour effects in various cancers. Previous studies have reported that Dox and Smac mimetics induce cell death mainly via the apoptotic pathway in tumour cells [16,17]. In this study, the apoptosis inhibitor z.VAD promoted cell death induced by SBP-0636457/Dox instead of inhibiting it (Figure 1(b)). In addition, a necroptosis inhibitor markedly reduced cell death caused by SBP-0636457/Dox (Figure 1(b)). Therefore, SBP-0636457/Dox induces necroptosis but not apoptosis in BC cells. This difference may be caused by the type of Smac mimetics and/or cell types since BC cells are sensitive to Smac mimetics and are more prone to necroptosis rather than apoptosis [18]. Further investigations are required to verify this hypothesis.

In this study, we measured the expression of regulatory proteins of cell death. All BC cells were found to express key necroptosis regulators, such as RIP1 and MLKL, but they did not express RIP3, a finding consistent with that of a previous study [18]. Using genetic silencing and pharmacologic inhibitors, RIP1 and MLKL were also found necessary for necroptosis induced by SBP-0636457/Dox in BC cells. The expression of RIP1 and MLKL was higher in BC tissues than in normal breast tissues [19]. Therefore, the application of SBP-0636457/Dox to induce necroptosis may be a potent strategy to induce cell death in BC cells.

Another vital finding of this study is that the constitutive secretion of TNF*α* is essential for necroptosis induced by SBP-0636457/Dox, which pharmacologically inhibits TNF*α* or genetic silencing of TNFR/IRF and protects BC cells from death. This finding is similar to that of previous studies, indicating that TNF*α*/TNFR signalling is required for cell death induced by Smac mimetics [18,20]. TNF*α*, a member of the TNF superfamily, can regulate cell death or survival after binding to its corresponding receptor TNFR1 [14]. Therefore, the role of TNF*α* in the tumorigenesis of BC remains controversial. On the one hand, TNF*α* can activate the mesenchymal stromal cells and thereby promote BC cell metastasis [21]. On the other hand, TNF*α* induces potent cytotoxic cell death in luminal (ER+) BC cell lines as characterised by the lack of A20 [22]. Furthermore, TNF*α* has been found to promote cell death induced by chemotherapy and radiotherapy in BC cells [23]. Therefore, TNF*α* is considered a double-edged sword in BC cells. In this study, SBP-0636457/Dox treatment promoted TNF*α* signalling and converted TNF*α* signalling into a prodeath stimulus in BC cells. Remarkably, using the CYT-6091 nanoparticle approach to deliver TNF*α* has been tested in a phase I clinical trial of patients with advanced-stage BC, and the results are encouraging [24].

Moreover, the role of NF-*κ*B signalling in cell death induced by SBP-0636457/Dox was also examined. The results suggest that both canonical and noncanonical NF-*κ*B promote necroptosis induced by SBP-0636457/Dox. Furthermore, genetic inhibition of either p65 or NIK only partially protected BC cells from SBP-0636457/Dox-induced cell death; however, inhibition of both p65 and NIK almost completely blocked necroptosis. This phenomenon may be caused by both canonical and noncanonical NF-*κ*B pathways that are involved in TNF*α* upregulation induced by SBP-0636457/Dox. This finding is consistent with that of previous studies, which also reported that both canonical and noncanonical NF-*κ*B pathways can regulate TNF*α* expression [25]. Considering that the NF-*κ*B pathway plays an essential role in both intrinsic and acquired resistance against endocrine therapy in patients with BC [26], the strategy of inducing necroptosis in patients insensitive to endocrine therapy should be examined.

However, this study has some limitations. First, the effects of SBP-0636457/Dox *in vivo* were not investigated owing to the limited time and funds. It would be interesting to test the combined treatment of SBP-0636457/Dox in a xenograft BC model. Second, inhibition of NF-*κ*B cannot completely inhibit TNF*α* upregulation. Therefore, some other pathways may compensate for NF-*κ*B inhibition. Further investigations are necessary to elucidate this finding.

## 5. Conclusion

SBP-0636457 and Dox combined treatment induces necroptosis in BC cells after inhibiting apoptosis. Mechanically, RIP1 and MLKL are required to promote necroptosis induced by SBP-0636457/Dox in BC cells. SBP-0636457/Dox activates the TNF*α*/TNFR signalling pathway, which is involved in inducing necroptosis. Furthermore, both canonical and noncanonical NF-*κ*B pathways are responsible for the upregulation of TNF*α* induced by SBP-0636457/Dox in BC cells. These findings suggest that cotreatment with SBP-0636457 and Dox is a promising strategy for the treatment of BC, especially in the case of insensitivity to apoptosis.

## Figures and Tables

**Figure 1:** Combined treatment with SBP-0636457 and Dox induced cell death by inhibiting apoptosis (a) BC cells were treated with different doses of SBP-0636457 for 24 (h), and cell death was measured. (b) BC cells were treated with SBP-0636457 (2 *μ*M), Dox (4 *μ*M), or SBP-0636457/Dox in the presence of z.VAD (20 *μ*M) or Nec-1 (10 *μ*M) for 24 h, and finally, cell death was measured. (c) Levels of indicated proteins were measured in BC cells. (d) BC cells were transfected with different siRNAs for 24 h, and finally, indicated proteins were measured. (e) BC cells were transfected with negative control siRNA (si-NC) or siRNAs against caspase-8 (si-C8) for 24 h, and cells were treated with or without SBP-0636457/Dox for another 24 h, and finally, cell death was measured. (f) BC cells were transfected with negative control siRNA (si-NC) or siRNAs against FADD (si-FD) for 24 h and treated with or without SBP-0636457/Dox for another 24 h, and finally, cell death was measured. Data were presented as the mean ± SD (^*∗*^*P* < 0.05; ^*∗∗*^*P* < 0.01).

**Figure 2:** RIP1 and MLKL are required for cell death induced by SBP-0636457/Dox in BC cells (a) BC cells were transfected with indicated siRNAs for 24 h, and RIP1 levels were measured. (b) BC cells were transfected with indicated siRNAs for 24 h and treated as indicated for another 24 h, and finally, cell death was measured. (c) BC cells were pretreated with RIP1 inhibitors (RIPA-56 10 *μ*M; GSK481 10 *μ*M) for 6 h and treated as indicated for another 24 h, and finally, cell death was measured. (d) BC cells were transfected with indicated siRNAs for 24 h, and MLKL levels were measured. (e) BC cells were transfected with indicated siRNAs for 24 h and treated as indicated for another 24 h, and finally, cell death was measured. (f) BC cells were pretreated with MLKL inhibitors (MLKL-IN-1 15 *μ*M; GW806742 × 10 *μ*M) for 6 h and treated as indicated for another 24 h, and finally, cell death was measured. Data were presented as the mean ± SD (^*∗*^*P* < 0.05; ^*∗∗*^*P* < 0.01).

**Figure 3:** TNF*α* signalling is required for cell death induced by SBP-0636457/Dox in BC cells (a) BC cells were treated with Dox, SBP-0636457, or their combination for 24 h, and TNF*α* levels in cell culture supernatants were measured by the ELISA. (b) BC cells were treated as described above, and TNF*α* mRNA levels were measured by RT-PCR. (c) BC cells were treated with z.VAD (10 *μ*M) or SBP-0636457/Dox/z.VAD in the presence or absence of Enbrel (5 *μ*M) for 24 h, and cell death was measured. (d) BC cells were transfected with the indicated siRNAs for 24 h, and TNFR levels were measured. (e) BC cells were transfected with the indicated siRNAs for 24 h and treated with z.VAD (10 *μ*M) or SBP-0636457/Dox/z.VAD for another 24 h, and finally, cell death was measured. (f) BC cells were treated with Dox, SBP-0636457, or their combination for 24 h, and IRF1 mRNA levels were measured. (g) BC cells were transfected with the indicated siRNAs for 24 h, and IRF1 protein levels were measured. (h) BC cells were transfected with the indicated siRNAs for 24 h and then treated with z.VAD (10 *μ*M) or SBP-0636457/Dox/z.VAD for another 24 h, and finally, cell death was measured. Data were presented as the mean ± SD (^*∗*^*P* < 0.05; ^*∗∗*^*P* < 0.01).

**Figure 4:** Both canonical and noncanonical NF-*κ*B pathways are involved in TNF*α* upregulation (a) BC cells were transfected with the indicated siRNAs for 24 (h), and p65 or NIK protein levels were measured. (b) BC cells were transfected with the indicated siRNAs for 24 h and treated with or without SBP-0636457/Dox/z.VAD for another 24 h, and finally, cell death was measured. (c) BC cells were treated with SBP-0636457/Dox/z.VAD for the indicated time, and finally, NIK expression was measured. (d) BC cells were transfected with the indicated siRNAs, and NIK expression was measured. € BC cells were transfected with the indicated siRNAs for 24 h and treated with or without SBP-0636457/Dox for another 24 h, and finally, mRNA levels of TNF*α* were measured. (f) BC cells were treated with different NF-*κ*B inhibitors (NG25 10 *μ*M; NIK SMI1 10 *μ*M; and DHMEQ 15 *μ*M) for 12 h and treated with or without SBP-0636457/Dox/z.VAD for another 24 h, and finally, cell death was measured. (e) TNF*α* mRNA levels were measured. Data are presented as the mean ± SD (^*∗*^*P* < 0.05; ^*∗∗*^*P* < 0.01).

**Table 1:** List of siRNA oligos for caspase-8, FADD, RIPK1, IRF1, MLKL, TNFR1, p65, NIK, and scramble negative control (si-NC).

Oligo	Sequence (5′-3′)
si-NC (negative control)	AACGUACGCGGAAUACUUCGA
si-caspase-8 #1	AAGAGTCTGTGCCCAAATCAA
si-caspase-8 #2	GACAAAGTTTACCAAATGAAA
si-FADD #1	TGGGCCGCTGCTTTGCGCTGG
si-FADD #2	AAGCAGAGAGGTGGAGAACT
si-RIPK1 #1	GAAAGAGTATTCAAACGAA
si-RIPK1 #2	GGGCTGATAACAGTGTTGT
si-IRF1 #1	CTGTGCGAGTGTACCGGATG
si-IRF1 #2	AGGCTACATGCAGGACTT
si-MLKL #1	TTCCAGATGCTAAGAAGAGA
si-MLKL #2	GTCCTAGTCCTGGGG
si-TNFR1 #1	TACGACTATGTTAACTAAATTG
si-TNFR1 #2	AGGCAACAGCTCAACCACA
si-p65 #1	GAACCTGGGAATCCAGTG
si-p65 #2	GCATCCAGACCAACAACAA
si-NIK #1	AGGGGCTGACGAGTCCA
si- NIK #2	CTCTTATCAACCGAAGACGA

**Table 2:** List of primers for RT-PCR.

Genes	Primers 5′-3′
TNF*α*	Forward: 5′-CGAGTGACAAGCCTGTAGCC-3′
	Revers: 5′-GTTGACCTTGGTCTGGTAGG-3′

GAPDH	Forward: 5′- GCAGGGGGGAGCCAAAAGGG-3′
	Revers: 5′-TGCCAGCCCCAGCGTCAAAG-3′

## Data Availability

Data are available on request.
